RETRACTED

# Bayes Clustering and Structural Support Vector Machines for Segmentation of Carotid Artery Plaques in Multicontrast MRI

**DOI:** 10.1155/2012/549102

**Published:** 2012-12-19

**Authors:** Qiu Guan, Bin Du, Zhongzhao Teng, Jonathan Gillard, Shengyong Chen

**Affiliations:** ^1^College of Computer Science, Zhejiang University of Technology, Hangzhou 310023, China; ^2^Department of Radiology, University of Cambridge, Hills Road, Cambridge CB2 0SP, UK

## Abstract

Accurate segmentation of carotid artery plaque in MR images is not only a key part but also an essential step for in vivo plaque analysis. Due to the indistinct MR images, it is very difficult to implement the automatic segmentation. Two kinds of classification models, that is, Bayes clustering and SSVM, are introduced in this paper to segment the internal lumen wall of carotid artery. The comparative experimental results show the segmentation performance of SSVM is better than Bayes.

## 1. Introduction

Cardiovascular diseases (CVDs) are the leading cause of death globally according to the recent statistics of the World Health Organization. Atherosclerosis, a kind of systematic inflammatory disease, is estimated to be responsible for CVDs to a great extent. Therefore, there are considerable interests in characterizing atherosclerotic plaques for proper treatment planning. Research in the past 20 years indicates that plaque vulnerability is very relative to its structure, such as the lumen condition, atherosclerotic components within the plaque [1–5]. 

As the fundamental step, artery wall should be segmented accurately. Meanwhile, explicit detection of wall is very important to locate each component inside the plaque correctly, which is also very significant for the subsequent procedures such as component analysis.

Automated analysis of plaque composition in the carotid arteries has been presented by many researchers. Different imaging techniques always bring out distinct characteristic of image, which will restrict different applicable approach to approach of segmentation. Among current standard imaging techniques in clinical, in vivo multicontrast MRI technique has been generally validated to be used to quantify the composition of plaque effectively [6]. Most segmentation methods based on this kind of imaging technique are generally based on manual extraction of numerous contours. Automatic segmentation not only makes the combination of different multicontrast-weighted MR Image possible, but also can further make full use of the advantages of different image to improve the accurate rate of classification of component within lumen. Other impressive experiments are also carried out by taking use of model-based clustering and fuzzy clustering [7], maximum-likelihood classifier and nearest-mean classifier [8], morphology-enhanced probability maps [9], and k-means clustering [10]. Most of these methods are based on voxel-wise statistical classification, and the manual analysis cannot be completely replaced by them. An automatic method which was used to segment the carotid artery plaques in CT angiography (CTA) [11] has potential to replace the manual analysis. Firstly, the vessel lumen was segmented. Subsequently, classifier was trained to classify each pixel. However, this algorithm is needed to be improved to deal with the multicontrast-weighted MR Image. Furthermore, in order to provide a more accurate and objective ground truth, a simultaneous segmentation and registration model [12] is necessary in registration. This method is an active contour model based on simultaneous segmentation and registration which is belong to mutual-information-based registration [13]. Therefore, researches concerning segmentation of plaques are essential.

RETRACTED

The paper is organized as follows. Significance of studying carotid artery plaque and current research contributions are briefly presented in Section 1.  Section 2 is mainly focus on describing major and special preprocessing such as ill-illumination uniforming and image registration. Two kinds of model used to segment the wall boundary are descried in detailed in Section 3.  Section 4 focuses on two algorithms to segment the lumen, and a conclusion and further work are presented in Section 5. 

## 2. Testing Image Set

The complete process of plaque analysis system is organized as below, which is composed of four modules. Firstly, carotid artery region should be separated from the original MRI image and then move on to the preprocessing parts including noise removal and illumination uniform. After that, the lumen and the outer wall in the images are obtained in turn. The latter operations are related with extracting and modeling essential plaque components, and mechanical analysis based on FSI (fluid-structure interaction) theory will be also introduced to estimate the risk extent of a plaque. The steps in Figure 1 will be discussed in detail in this paper.

### 2.1. Acquisition of Testing Image Set

Images used in our research are acquired by a MRI scanner named GE SIGNA. Taking Figure 2(a) for instance, it can be found that carotid arteries marked by two rectangles are closely surrounded by other tissues as muscles, fat, bones, and other vessels in the 512 mm × 512 mm MRI image. In order to handle carotid artery alone as shown in Figure 2(b), small ROI of each artery region should be firstly segmented from the original scanning image by picking out the artery centroid which size is 81 mm × 81 mm. The reduction of interested region effectively avoids disturbing from other tissues and also improves the computing speed. 

RETRACTED

The detail of MRI acquisition has already been published in [14]. Briefly speaking, patients undergo high resolution MRI of their carotid arteries in a 1.5 Tesla MRI system (named as Signa HDx GE Healthcare, Waukesha, WI, USA) with a 4-channel phased-array neck coil (named as PACC, Machnet BV, Elde, The Netherlands). Artifact resulted from movement is minimized by using a dedicated vacuum-based head restraint system (VAC-LOK Cushion, Oncology Systems Limited, UK). It is used to fix the head and neck of patient in a comfortable position to avoid occurrence of artefact. After an initial coronal localizer sequence is sampled and tested, 2-dimensional (2D) axial time-of-fight (TOF) MR angiography is performed to identify the location of the carotid bifurcation and the region of maximum stenosis. Axial images are acquired through the common carotid artery 12 mm (4 slices) below the carotid bifurcation to a point 12 mm (4 slices) distal to the extent of the stenosis identified on the TOF sequence. This kind of method ensures that the whole region of carotid plaque is completely imaged.

To describe the characteristic of different MRI sequence, the following parameters are used: T1 weighted (repetition time/echo time: 1  ×  RR/7.8 ms) with fat saturation, T2 weighted (repetition time/echo time: 2  ×  RR/100 ms) with fat saturation, proton density weighted (repetition time/echo time: 2  ×  RR/7.8 ms) with fat saturation, and short-time inversion recovery (repetition time/echo time/inversion time: 2  ×  RR/46/150 ms). The window of view of each MR image is 10 cm × 10 cm, and size of data matrix is 512 × 512. The spatial resolution achieved of each pixel is 0.39 mm × 0.39 mm.

In Figure 2(a), two small ROIs marked by red rectangles are carotid arteries each size of RIO is 81 mm × 81 mm. Figure 2(b) is the amplified images of these two areas.

### 2.2. Preprocessing

Due to the inhomogeneity of coil, the intensity of each image should be adjusted to be relative uniform to obtain relative consistent gray scale for the subsequent segmentation based on clustering. The region (14 mm × 14 mm), which lies in the center of the vessel, is selected as the interesting region. The contrast of the image is increased by a linear transformation,

(1) $$\begin{array}{c} u_{1}=\frac{u_{0}-m}{M-m}\times 255, \end{array}$$

where *u*_0_ is the initial intensity, *u*_1_ is adjusted intensity, and  *M*  and  *m*  are the maximum intensity and minimum intensity of the original image. The adjusted results of intensity uniform are shown in Figure 3.

RETRACTED

### 2.3. Image Registration

According to the characteristics of MR image, the contour of lumen is clearly presented in the sequence of T1 which is blood suppressed for short. In Figure 4, mark two feature points in images (a) and (b) as red points. Normally, the luminal bifurcation and narrowest location are selected as marking points for registration.

Generally speaking, the image is indistinct as shown in Figure 4. Therefore it is very difficult to mark feature points in some images. In order to deal with this problem, the registration method proposed in this paper is based on prior-constrained segmentation of carotid artery under DOG scale space. As seen from the name, the segmentation algorithm implies two parts. First, inspired by SIFT algorithm, the advantage of difference of Gaussian (DOG) scale space is introduced to catch the edges that seem ambiguous in the original image scale, which is the scale derivative of Gaussian scale space along the scale coordinate. Second, given a simple prior knowledge that the artery wall is near round, a given thickness of carotid artery wall is set to restrict the searching area. Prior shape is critical information for external wall segmentation. The steps to get the wall boundary are shown in Figure 5.

Then through minimizing the energy function using a gradient flow, we can achieve the goal of simultaneous segmentation and registration [12]. On the one hard, this new method can reduce the influence of noise on the original images and lead to improved registration, on the other hand it also can improve the precision segmentation, especially for segmentation the blurred images.

Given two images *I*_1_ and *I*_2_; *C*_1_ is the object contour of *I*_1_, and *C*_2_ is the object contour of *I*_2_. Establish mapping *C*_2_ = *g*(*C*_1_). The steps of simultaneous segmentation and registration method are listed as follows.

**Step 1**

Initialize *C*_1_,  *g*, and *C*_2_.

**Step 2**

Optimize the registration parameters to obtain the optimal mapping function  *g*.

**Step 3**

Evolute *C*_1_ to obtain the optimum partition line of the current image *I*_1_, and obtain the optimal split line of the current image  *I*  by *C*_2_ = *g*(*C*_1_).

**Step 4**

Reach the maximum number of iterative steps, or before and after the two results of the iteration are less than the threshold value then the algorithm stops, ended; otherwise turn to Step 2.

## 3. Modelling

 To compare the results of different algorithm of modeling, two kinds of model which are based on Bayes classification algorithm and SSVM (structural support vector machines) are carried out in this paper.

RETRACTED

### 3.1. Building of Training Set

From MRI slices with matching histological slices, slices 12 and 25 are selected to generate the training set for segmentation. Images of those two slices are manually segmented based on registered histological results and relative intensity. A total of 549 pixels (each pixel contains 4 densities representation with total 4 different contrast weight) are selected randomly in the investigation. From these segmentation results, each pixel is determined to belong to one of the 4 issue types including lipid (denoted as *Z*_1_), normal issue (denoted as *Z*_2_), calcification (denoted as *Z*_3_), and others (including lumen or outer issue, denoted as *Z*_4_). The training set is used to generate the probability function which is used to determine the probability of tissue type of each pixel in the model based on Bayes classification.

### 3.2. Model Based on Bayes Classification

The most important part of the segmentation algorithms is to determine the probabilities of each pixel. These probabilities represent the likelihood that the tissue of the pixel at the current location is lipid, calcification, normal issue, or others.

Maximum classifier is used to determine which issue type the pixel belongs to.  Figure 6 gives the flow-chart of our maximum decision probability functional classifier. Where $\vec{I}$ is one pixel of multicontrast weighted MR images transformed by preprocessing, $g_{i}(\vec{I})$ is the decision function, and $P(Z_{i}|\vec{I})$ is class-conditional probability density function (pdf). By comparing values of four functions, if $g_{i}(\vec{I})$ is the maximum probability value of one pixel, then pixel $\vec{I}$ belongs to *Z*_*i*_ and is labeled *i*.

### 3.3. Model Based on SSVM

Recently, structured prediction has already attracted much attention, and many approaches have also been developed based on it. Structured learning is one of the main approaches of structured prediction, which not only studies the problems with well-structured inputs and outputs but also reveals strong internal correlations. It is formulated as the learning of complex functional dependencies between multivariate input and output representations. Structured learning has significant impact in addressing important computer vision tasks.  Figure 7 gives the flowchart of SSVM to obtain gray information. The flowchart of the iterative training of SSVM is given in Figure 8.

## 4. Comparison

The results of segmentation of slices 28 and 34 MR images based on Bayes and SSVM are illustrated in Figure 9.

As seen in Figure 9, the segmentation result in term of classification algorithm reveals that the performance of SSVM is much better than that of Bayes due to the former including structural information, and smoothing effect of segmentation of SSVM is also obvious. 

RETRACTED

The results presented by image are inadequate to make evaluations. Here a parameter named misclassification rate is defined to judge the accuracy of each algorithm. 

In the experiment of this paper, a selected slice MR image is corrupted by global intensity varying from 20% to 40% and adding 1%–9% noise. Misclassification rate, an evaluating criterion, is defined as the ratio of misclassified pixels to total number of pixels of this class. It is formulated as (2) as follows:

(2) $$\begin{array}{c} e\left(i\right)=\frac{fp+fn}{n}, \end{array}$$

where *e*(*i*) is the misclassification rate of tissue *i*;  *fp*  is the false positive responses (pixel belongs to tissue  *i* but is classified as other tissues);  *fn*  is the false negative responses (pixel does not belong to tissue *i* but is classified as tissue type *i*);  *n*  is the total number of pixels of tissue type *i*. 

The misclassification rate of lumen obtained by Bayes and SSVM algorithm is listed in Table 1. From the statistics shown in Table 1, it can be seen that the misclassification rate caused by SSVM is much lower than that of Bayes. That stands for the performance of SSVM outperforms that of Bayes, especially while the level of noise is higher.

## 5. Conclusion

To summarize, the work in this paper is focus on the first several steps of carotid artery plaque analysis, including preprocessing of MR image, model-based segmentation of lumen, plaque, and external wall. Two kinds of model, Bayes and SSVM, are separately constructed and applied to the detection of internal wall. Receivable boundaries can be both obtained by two algorithms, the results of experiment shows the segmentation performance of SSVM is better than that of Bayes, especially, while the level of noise in image is higher.

But there are still some improvements need to be done in the future to break the limitations of the current work. Firstly, improve Bayes to better performance by increasing structural information. Secondly, introduce sequence image tracking technique in research to improve the performance of human interaction to specify the center of lumen. Further effort should focus on estimation of artery location in each MRI slice and take advantage of information gained from previous slice to pick out the artery centroid of current image. Moreover, several other algorithms need to be testified and compared with them when dealing with plaques.

## Figures and Tables

**Figure 1:** Flow of operations.

**Figure 2:** ROI extraction: (a) original MRI image, (b) extracted images.

RETRACTED

**Figure 3:** Preprocessing of selected slices of MR images: (a) a set of original images, (b) resultant images after contrast normalization.

**Figure 4:** Handle marking points for registration: (a) MR images, (b) manual outline, (c) result of registration.

**Figure 5:** Flowchart of multiscale PCA.

**Figure 6:** Flowchart of maximum decision probability functional classifier.

**Figure 7:** Flowchart of SSVM to obtain gray information.

**Figure 8:** Flowchart of the iterative training of SSVM.

**Figure 9:** Two segmentation results of selected slice using multicontrast MR images: (a) testing MR images; (b) automatic segmentation results of Bayes classifier; (c) automatic segmentation results of SSVM process.

**Table 1:** Misclassification rate of lumen for Bayes and SSVM.

Noise	Misclassification rate	
	Bayes	SSVM
1%	3.5	2.6
3%	5.3	4.8
5%	6.5	6.3
7%	10.6	8.5
9%	16.9	9.6
